The article "The Application of Artificial Intelligence Technology in the Asset Management of Start-Ups in the Context of Deep Learning" was published in 2022. Journal: Comput Intell Neurosci.

# The Application of Artificial Intelligence Technology in the Asset Management of Start-Ups in the Context of Deep Learning

**DOI:** 10.1155/2022/1756470

**Published:** 2022-05-05

**Authors:** Qi Fu, Xiaotong Li

**Affiliations:** ^1^Department of International Finance, Shanghai Lixin University of Accounting and Finance, Shanghai 200000, China; ^2^Department of Finance and Business Economics, University of Macau, Macau 999078, China

## Abstract

With the coninuous improvement and development of artificial intelligence (AI) technology, this technology has been used in the asset management of companies. To improve the asset management level of Chinese start-ups, firstly, back-propagation neural network (BPNN) has been studied in depth, and an evaluation system of the company's asset quality has been established. Secondly, the BPNN is integrated with the evaluation indicators of asset quality, and an evaluation model of asset quality based on BPNN is constructed. Next, start-up A is taken as the experimental object; the evaluation score of the asset quality of A company is input into the model, which proves that there is still a certain gap between the asset management level of start-ups and mature companies. Finally, to find out the problems of the company's asset quality, the traditional financial analysis method is used to carry out a specific microanalysis of the evaluation indicators of its asset quality. In view of the existing problems, suggestions are put forward for prudent investment, improve inventory operation efficiency, increase investment in R&D and innovation, improve the quality of sales outlets, and increase the proportion of high-quality intangible assets. The asset quality evaluation system for start-ups established here includes 19 evaluation indicators. The BPNN-based asset quality evaluation model selects 5 mature companies in the same industry as sample companies. The scores of the evaluation indicators of asset quality of the 5 sample companies in the past three years are normalized and input into the model. The model contains 19 nodes of the input layer, 39 nodes of the hidden layer, and 1 node of the output layer. The target error rate is 0.001, the learning rate is 0.1, the number of training times is 1000, and the training function is the trainlm function. This research has a certain reference for the application of AI technology in the asset management of start-ups.

## 1. Introduction

In recent years, with the rapid development of artificial intelligence (AI), today's society is paying more and more attention to technological innovation, functional integration, and value enhancement through AI. The AI AlphaGo has defeated the human Go master. Traders and other positions in financial institutions on Wall Street are also being largely replaced by AI [1]. At this stage, with the continuous improvement and development of AI technology, it has gradually become popular in people's lives. To a large extent, this makes people's lives more intelligent, and meanwhile, it greatly promotes the development of enterprise asset management. Assets, as the material basis for the survival of enterprises, are also the material guarantee for enterprises to win in the market competition. During the entire existence of an enterprise, the quality of the assets determines the quality of the enterprise's survival, which directly affects the success or failure of the enterprise's production and operation. Therefore, more attention is paid to enterprise assets management.

The article "The Application of Artificial Intelligence Technology in the Asset Management of Start-Ups in the Context of Deep Learning" was published in 2022. Journal: Comput Intell Neurosci.

With the development of the times, the content of assets has changed. Human resources, innovation capabilities, brand value, and so on are also valuable resources of enterprises and play a vital role in enterprise assets. However, the measurement method of such assets is still an unsolved problem [2]. Ali et al. (2021), to improve the accuracy of asset quality evaluation of banks, when constructing an index system of the asset quality evaluation, tried to combine the G1 weighting method and the mean square error (MSE) to determine the index weight. Thereby, a scientific comprehensive evaluation model based on the weighting method was established, and an empirical analysis was carried out on the asset quality level of nine commercial banks [3]. Zheng (2021) proposed a new hybrid wavelet kernel function and introduced it into the support vector machine (SVM) to innovate the asset quality evaluation model. Finally, the model was used to detect the asset quality anomaly of A-share listed manufacturing enterprises. The results showed that the recognition rate of the model for abnormal samples had been greatly improved [4]. Judging from the existing research, people focus on mature companies or listed companies, and few people pay attention to start-ups. Therefore, this research will focus on improving the asset management level of start-ups. Cai et al. (2019), to improve the coordination between supply chain node enterprises and ensure the normal operation of the supply chain, established a supply chain risk assessment model using BPNN. The results demonstrated that BPNN had unique advantages in solving highly nonlinear problems such as risk assessment, and the evaluation model could provide effective decision support for supply chain risk management [5]. Therefore, this research will also evaluate the asset quality of startups by establishing a BPNN model to provide effective decision support for them and improve their asset management level.

The article "The Application of Artificial Intelligence Technology in the Asset Management of Start-Ups in the Context of Deep Learning" was published in 2022. Journal: Comput Intell Neurosci.

To improve the asset management level of Chinese start-ups and solve the problems encountered by start-ups in the development, firstly, back-propagation neural network (BPNN) is studied in depth. Secondly, an evaluation indicator of asset quality for the start-ups is established, and an evaluation model of asset quality based on BPNN is constructed. Finally, start-up A is taken as the research object. Through the evaluation model of asset quality based on BPNN, the specific situation of the company's asset quality is deeply explored, and analysis and suggestions are made on the exploration results. This research has a certain reference for the application of AI technology in the asset management of start-ups.

## 2. BPNN and Evaluation Model of Asset Quality

### 2.1. BPNN

Since the development of artificial neural network (ANN), a variety of algorithms have been bred, and BPNN is a typical learning algorithm, which is characterized by forward propagation of information and back-propagation of errors, to carry out the self-learning process of the network. The neurons of BPNN are arranged hierarchically, including input layer, hidden layer, and output layer. The neurons of the same layer are not connected to each other; only the neurons of the adjacent upper and lower layers can be connected to each other. BPNN can generate different output information by inputting different input data to satisfy all training sets as far as possible [6]. Its structure diagram is shown in Figure 1.

When BPNN performs operations, the transfer function between neurons is a sigmoid differentiable function. The feature of this function is that it can complete any form of nonlinear mapping between the input layer and the output layer. Therefore, it endows the BPNN with absolute advantages in solving the problems of data classification, pattern recognition, and risk assessment [7–9].

After the input layer receives the input data, it propagates to the node of the hidden layer. After the neuron of the hidden layer receives the data, after the operation of the sigmoid-type activation function, the calculated data is transmitted to the node of the output layer. Finally, the output result is obtained. The sigmoid function includes two forms, namely, log-sigmoid function and tan-sigmoid function [10]. The expression of the log-sigmoid function is shown as follows:

(1) $$\begin{array}{c} f\left(x\right)=\frac{1}{1+e^{-x}}. \end{array}$$

The expression of the tan-sigmoid function is as follows:

(2) $$\begin{array}{c} f\left(x\right)=\frac{1-e^{-x}}{1+e^{-x}}. \end{array}$$

In the process of data transmission, there is also the learning process of neural network (NN), which is an important operation process for BPNN to complete self-learning and objective weighting. The process mainly includes forward propagation and back-propagation. During forward propagation, the input data is transmitted from the input layer to the hidden layer and then propagated to the output layer after data processing. In this process, the state of neurons in each layer only affects the neurons in the next layer. If the result obtained by the output layer does not meet the previous limited error rate, then back-propagation will be performed, and the error signal propagates in the reverse direction of the path in the forward propagation. In this process, the connection weights determined between each neuron are adjusted one by one. This process of forward and backward propagation is continuously iterated, and finally, the error rate of the output results is within a limited range [11, 12]. The specific process is shown in Figure 2.

The article "The Application of Artificial Intelligence Technology in the Asset Management of Start-Ups in the Context of Deep Learning" was published in 2022. Journal: Comput Intell Neurosci.

### 2.2. Evaluation Indicators of Asset Quality

The characteristics of asset quality are divided into five aspects: existence, turnover, profitability, structure, and liquidity. (1) The existence of assets is a feature used to measure the authenticity of assets, which can reflect the existence of assets in the company. Assets can be regarded as resources owned and controlled by companies only if they can be actually applied in the process of company operation, and such assets are real assets [13]. (2) The characteristics of turnover reflect the efficiency of asset creation benefits and are generally reflected by indicators related to the turnover rate. Assets need to be utilized to play a role, and the completion of a cycle of circulation can bring economic benefits. Therefore, on the one hand, the turnover rate reflects the efficiency of the income brought by assets participating in the operation of the company, and on the other hand, it reflects the level of the company's management ability [14]. (3) Profitability is the core indicator for examining companies, and it is also a significant feature to measure asset quality. Whether other qualities of assets show upward or downward trends, they will be clearly reflected in the quality of earnings, and profitability is also the most direct feature to evaluate asset quality [15]. (4) Companies need various assets to meet the complex needs of their production and operation, and various assets will inevitably form different asset structures. The asset structure is reflected by the type of assets and the ratio between each asset. Different asset structures reflect different strategic layouts of companies as well as different risks. The asset structure needs to be scientifically arranged on the basis of considering the development strategy of the company. A reasonable asset structure can promote the stable operation of the company according to the business strategy and reduce the comprehensive capital cost rate and financial risk of the company [16]. (5) Liquidity is a feature that measures the ability of an asset to obtain cash. Only by having sufficient cash flow can ensure the smooth progress of each operation cycle of the company, and the company can carry out a new round of investment as scheduled. The liquidity of assets is an upgrade requirement for the profitability of assets. If the assets have a strong ability to obtain income, but the income cannot be actually used by the company and put into production and operation, the quality of the income obtained by the assets will be poor, and the profitability of the asset needs to be further investigated by using the liquidity [17].

The article "The Application of Artificial Intelligence Technology in the Asset Management of Start-Ups in the Context of Deep Learning" was published in 2022. Journal: Comput Intell Neurosci.

For start-ups, it has the following three outstanding characteristics: (1) The proportion of fixed assets is large. In the early stage of the company's establishment, a large number of production operations are required, so more funds will be invested in fixed assets such as machinery and equipment. And fixed assets are the main fixed costs of start-ups. They have the characteristics of strong specificity and poor liquidity. Therefore, the existence, structure, and turnover of asset quality are very important to the home appliance industry, and these asset quality characteristics need to be considered when selecting relevant indicators. (2) There are few product types and the process is fixed. The main products of start-ups are usually fixed to a few types. At the same time, due to the high cost of production equipment, it is difficult to update quickly, resulting in a fixed process. When large-scale production is carried out, if the products on the assembly line do not enter the circulation link in time, a large amount of working capital will be occupied, and the cash flow of the company will be at risk of rupture. Therefore, in the evaluation of asset quality, indicators that reflect the inventory level and turnover rate of companies should be selected [18]. (3) Lack of core technology and poor product innovation capability: since the production technology and core technology of start-ups lag behind mature companies, their product innovation capabilities are relatively poor. It is necessary to invest more R&D and continuously carry out technological reforms. Therefore, the selection of evaluation indicators of asset quality also needs to be able to reflect the situation of intangible assets of companies [19, 20]. According to the characteristics of start-ups, the evaluation indicators of asset quality are formulated, and the specific indicators selected are shown in Figure 3.

The article "The Application of Artificial Intelligence Technology in the Asset Management of Start-Ups in the Context of Deep Learning" was published in 2022. Journal: Comput Intell Neurosci.

Different evaluation indicators measure different aspects of asset quality, which have different meanings and different calculation methods, which lead to different calculation results for each indicator and large differences in the evaluation standards of each indicator. Different dimensions are formed between them, which will reduce the accuracy of the evaluation results of the model and increase the computing time of the model [21]. To unify the different dimensions between the indicator values and solve the problem of comparability of the indicators, it is necessary to normalize the data in advance so that the data are all in a uniform order of magnitude, which is convenient for the model to run and finally get the comprehensive evaluation results. When establishing the asset evaluation model of the BPNN, the premnmx(P) function in MATLAB software is used for normalization. The specific calculation is shown as follows:

(3) $$\begin{array}{c} P_{n}=\frac{2*\left(P-\text{min}p\right)}{\left(\text{max}p-\text{min}p\right)}-1. \end{array}$$

In (3), *P* is the original input data, that is, the result obtained after calculation according to the evaluation indicator of the asset quality. max*p* and min*p* are the maximum and minimum in *P*, respectively, and *P*_*n*_ is the normalized input data.

### 2.3. Construction of Evaluation Model of the Asset Quality Based on BPNN

To establish an evaluation model of the asset quality based on BPNN, it is necessary to objectively evaluate the asset quality of the sample companies in advance and take the evaluation result as the expected output value of the model. On this basis, the input and output data pairs are formed, and the “data pairs” are used to learn and train the model. The error rate between the actual output and the expected output is used to judge whether the model is successfully established [22]. The entropy weight method is used to determine the expected output of the model. The specific calculation process is as follows.

(1) *Normalization of Original Data*. The collected evaluation indicator data of 5 mature companies in the same industry in the past three years is used as the original data to form the original matrix X={x_ij_}, and the original data is normalized. At this time, the normalization needs to further distinguish the properties of each indicator and normalize the indicators of different properties respectively. For the cost indicator data (the smaller, the better the data), the following equation is used for normalization:
  (4) $$\begin{array}{c} v_{ij}=\frac{x_{ij}-\text{min}\left(x_{j}\right)}{\text{max}\left(x_{j}\right)-\text{min}\left(x_{j}\right)}. \end{array}$$
For the benefit indicator data (the bigger, the better the data), the followingequation is used for normalization:
  (5) $$\begin{array}{c} v_{ij}=\frac{\text{max}\left(x_{j}\right)-x_{ij}}{\text{max}\left(x_{j}\right)-\text{min}\left(x_{j}\right)}. \end{array}$$
In (4) and (5), *x*_*ij*_ represents the *j*th indicator data of the *i*th company. *v*_*ij*_ shows the normalized value of *x*_*ij*_, max(*x*_*j*_) means the maximum value in the *j*th indicator data, and min(*x*_*j*_) refers to the minimum in the *j*th indicator data. According to the meaning of the evaluation indicators, the properties of each evaluation indicator are finally determined, as shown in Figure 4.
In Figure 4, due to the different business strategies of different companies, it is impossible to clearly determine the specific properties of the fixed asset ratio and asset-liability ratio. However, whether these two evaluation indicators are too large or too small will bring risks to the company. Therefore, the industry average is used as the standard value [23, 24].
(2) The proportion of each data in all data columns is calculated, as shown in the following equation:
  (6) $$\begin{array}{c} P_{ij}=\frac{V_{ij}}{\sum_{i=1}^{m}V_{ij}}. \end{array}$$
In (6), *P*_*ij*_ is the proportion of the feature of the *i*th evaluation object in the *j*th indicator, and *m* is the number of sample companies.
(3) The entropy value of the indicator is calculated, as shown in the following equation:
  (7) $$\begin{array}{c} e_{j}=-\frac{1}{\text{ln}\left(m\right)}\overset{m}{\underset{i=1}{\sum }}P_{ij}\text{ln}\left(P_{ij}\right). \end{array}$$
In (7), *e*_*j*_ expresses the entropy value of the *j*th indicator.
(4) The coefficient of variance of the indicator is calculated. According to the concept of entropy, when the amount of information increases, the entropy decreases. Therefore, for an indicator *D*_*j*_, the smaller the difference in the normalized value *v*_*ij*_ of the indicator, the larger the *e*_*j*_, and the less the amount of information contained in the indicator. The value of *e*_*j*_ is 1 when the values of the *j*th indicator of the evaluated object are all equal [25]. The difference coefficient of the indicator is calculated as shown in the following equation (8):
  (8) $$\begin{array}{c} d_{j}=1-e_{j}. \end{array}$$
In (8), *d*_*j*_ is the difference coefficient of the *j*th indictor; the larger *d*_*j*_, the greater the amount of information provided by the indicator, and a greater indicator weight should be given.
(5) The entropy weight of the indicator is determined, as shown in the following equation:
  (9) $$\begin{array}{c} w_{j}=\frac{d_{j}}{\sum_{j=1}^{n}d_{j}}. \end{array}$$
In (9), *w*_*j*_ represents the weight of the *j*th indicator, and *n* denotes the total number of indicators. In the end, the weights of each evaluation indicator for each year of mature companies in the same industry in the past three years are calculated as shown in Figure 5.
(6) The comprehensive score of the asset quality of the sample companies is calculated, as shown in the following equation:
  (10) $$\begin{array}{c} z_{i}=\overset{n}{\underset{j=1}{\sum }}W_{j}V_{ij}. \end{array}$$

In (10), *z*_*i*_ indicates the comprehensive score of asset quality of the *i*th company. The comprehensive score of asset quality of the five mature companies in the same industry in each year is shown in Figure 6.

The article "The Application of Artificial Intelligence Technology in the Asset Management of Start-Ups in the Context of Deep Learning" was published in 2022. Journal: Comput Intell Neurosci.

Through the progressive average method, the comprehensive score of the company's asset quality is graded. The standard of grade classification is shown in Figure 7.

The results of these grades classification will be used as the expected output value when training the NN. The expected output value is compared with the actual output value judged by the established BPNN, and the network structure and network parameters of the optimal NN are selected according to the size of the error rate.

The input layer is used to accept external input data. The number of nodes in the input layer is determined by the specific problem that the NN needs to solve. The number of nodes is equal to the number of types of input data in the actual problem. A total of 19 evaluation indicators are selected when determining the evaluation indicator system of asset quality, so the number of nodes in the input layer of the BPNN established this time is 19. The output result of the output layer is any value within the range of the grade value, and the output result is divided into different evaluation grades by rounding. Hence, it is finally determined that the output layer of the model has only one node. For the number of nodes in the hidden layer, it is based on Kolmogorov's theorem and combined with the experimental method to determine the number of nodes in the hidden layer. After many experiments, it is finally determined that the number of nodes in the hidden layer is 39, and the correct rate at this time is 98%.

The sigmoid-type differentiable function is generally determined between the neurons in the hidden layer of the BPNN because this function can complete any nonlinear mapping, ensuring that the network can fully reflect all the data characteristics. Through experiments, it is found that when evaluating asset quality, the transfer function between the input layer and the hidden layer using the tan-sigmoid function is more accurate than the log-sigmoid function. Meanwhile, since the expected output value has been obtained, the output result will be any value between (0, 5). The purelin function is used as the transfer function between the hidden layer and the output layer so that the output result can take any value [26–28]. Accordingly, the tan-sigmoid function, the sigmoid function, and the purelin function are determined as the transfer functions of the input layer, the hidden layer, and the output layer, respectively.

The article "The Application of Artificial Intelligence Technology in the Asset Management of Start-Ups in the Context of Deep Learning" was published in 2022. Journal: Comput Intell Neurosci.

The standard BP learning algorithm has the defects of easily falling into local minimum value and slow convergence speed. After using various common optimization learning algorithms to train the NN this time, it means that the trainlm function has fast convergence speed, strong stability, and small result error. It is more suitable for the construction of this evaluation model. The performance of the trainlm function will deteriorate with the increase of the network size, and the number of samples data of this model is small, so it is more conducive to the trainlm function to maintain the best performance, so the trainlm function is finally selected as training function of the model.

After the training function is determined, various parameters in the function need to be determined. The determination of the parameters is mainly determined according to the actual situation, such as the amount of model data, the complexity, and the required stability. “epochs” is used to limit the maximum training times of the network. When the number of training times reaches the epochs value, the training will stop. This parameter is generally determined according to the scale of the model. Since the number of the input data of this model is small, the scale of the model is small, and the epochs are finally determined to be 1000 times; “goal” is used to limit the error value of the target. If the error reaches the limit value during training, it means that the accuracy of the model has reached the expected value, and the training will stop. To improve the accuracy of the results, the error rate of this model is determined to be 0.001. “lr” (learning rate) is the limited parameter of the training speed. When the training speed is too fast, the network instability will increase. If the training speed is too small, the training time will be too long. After repeated experiments, it is determined that the training time and stability are better when the lr of the model is 0.1.

The article "The Application of Artificial Intelligence Technology in the Asset Management of Start-Ups in the Context of Deep Learning" was published in 2022. Journal: Comput Intell Neurosci.

## 3. Experimental Results and Analysis

### 3.1. Experimental Results

The scores of the evaluation indicators of the asset quality of the five sample companies in the past three years are normalized and input into the model. Therefore, the training samples consist of 15 pairs of input data. The training times and training results are shown in Figure 8.

The financial data of start-up A is calculated according to the determined evaluation indicator system of asset quality, and normalized, and then the normalized data is input into the trained BPNN evaluation model. The original input data of the evaluation model of asset quality of Company A since its establishment one year is shown in Figure 9.

In Figure 9, the ordinate is the original value of the asset quality evaluation of each index, and the abscissa is the code of each index. The original data is input into the trained BPNN model, and finally the output result of Company A is 3.1125, and the grade is divided into 4 levels, indicating that there is still a certain gap between the start-up A and other mature companies in the same industry in evaluation of asset quality. To find out the problems existing in the asset quality of the company, the traditional financial analysis method is used to carry out a specific and microscopic analysis of its evaluation indicator of asset quality.

### 3.2. Results and Analysis

To complete the vertical comparison of indicators between companies, the various evaluation indicators of asset quality of Company A are compared with those of mature companies in the same industry. To reflect the level of Company A's relevant indicators in the industry, the industry average is also added to the data comparison. The comparison of asset existence is as shown in Figure 10.

In Figure 10, the ratio of nonperforming assets and asset impairment ratio of Company A are higher than those of mature companies in the same industry. This is because Company A is in the start-up stage, with a large investment in decoration fees, advertising fees, and other expenses and inventory turnover rate. The lower bad debt loss ratio is due to less investment in new development projects and fewer customers participating in existing projects. With the increase in the number of customers and new projects in the future, the bad debt loss ratio will be close to the industry average.

The comparison of asset turnover is shown in Figure 11.

In Figure 11, the ordinate is the score of each index, and the abscissa is the code of each index. Only the accounts receivable turnover rate of Company A is better than that of mature companies in the same industry, and the turnover rate of other assets is relatively low. This is also because Company A is a start-up with fewer customers, less total assets, and most of them are fixed assets. In the early days of Company A, the output value is low, which also leads to a low turnover rate of fixed assets.

The article "The Application of Artificial Intelligence Technology in the Asset Management of Start-Ups in the Context of Deep Learning" was published in 2022. Journal: Comput Intell Neurosci.

The comparison of asset liquidity is shown in Figure 12.

In Figure 12, Company A's liquidity rate of total asset and operating profit liquidity rate are lower than those of mature companies in the same industry. This is because Company A, as a start-up, lacks core technologies. Although it has more fixed assets, its productivity is low, and the core components of its products are basically dependent on other companies, resulting in high costs. So, it is weaker than mature companies in the same industry in terms of asset liquidity.

The comparison of asset profitability is shown in Figure 13.

In Figure 13, as a start-up, Company A has less gap in asset profitability than mature companies in the same industry. The main reason is that although Company A has lower sales, its total assets are smaller than those of mature companies in the same industry. The sales area is smaller, so the transportation cost will be much lower, which eventually leads to Company A's, although it is a start-up, profitability being less than that of mature companies in the same industry. If the core technology is improved, the profitability will increase greatly.

The comparison of asset structure is shown in Figure 14.

In Figure 14, the ratio of fixed asset of start-up A is higher than that of mature companies in the same industry. This is because Company A, as a start-up, its main assets are mainly fixed assets, and the high proportion of fixed assets means that the company risk is high. The ratio of intangible assets of Company A is much lower than that of mature companies in the same industry. Due to the lack of core technologies of Company A, resulting in fewer awards and patents, the ratio of current assets of Company A's inventory is slightly higher than that of mature companies in the same industry. The lower the current asset ratio of the inventory, the better; that is, the less inventory, the more reasonable the asset structure of the company. The current asset ratio of Company A's inventory is still slightly higher based on weak productivity, which means that the company's sales need to be improved.

### 3.3. Advice to Company A

To sum up, to enable Company A to develop steadily, the following suggestions are put forward: (1) Invest cautiously, make rational decisions on investment strategies, and pay attention to the provision for asset impairment. (2) Improve the efficiency of inventory operation, determine production based on sales, attach importance to marketing strategies, and improve the use efficiency of idle funds. (3) Keep up with market demand, continuously launch new products, increase investment in research and development (R&D) and innovation, promote the progress of production technology, and strive to develop unique patented technologies of the company. (4) Improve the growth quality of offline outlets, select areas with higher income growth rates to add new outlets, regularly check the sales status, increase efforts to develop a series of products for the mass market, and expand the consumer groups of the products. (5) Improve the proportion of intangible assets of companies with high quality, increase investment in R&D, and appropriately adjust the proportion of fixed assets on the basis of considering the overall economic form so that the scale of company assets matches the number of production equipment and give full play to the production potential that the company should have.

The article "The Application of Artificial Intelligence Technology in the Asset Management of Start-Ups in the Context of Deep Learning" was published in 2022. Journal: Comput Intell Neurosci.

## 4. Conclusion

To improve the asset management level of start-ups, this research takes start-up A as the research object. Firstly, 19 evaluation indicators of asset quality are formulated based on the five characteristics of asset quality of existence, turnover, profitability, structure, and liquidity. Secondly, the BPNN is integrated and an evaluation model of asset quality is constructed. In the model, 5 mature companies in the same industry are selected as sample companies, and the scores of the evaluation indicators of asset quality of the 5 sample companies in the past three years are normalized and input into the model. The model contains 19 nodes of the input layer, 39 nodes of the hidden layer, and 1 node of the output layer. The target error rate is 0.001, the learning rate is 0.1, the number of training times is 1000, and the training function is the trainlm function. Then, the evaluation score of the asset quality of Company A is input into the model, and the output result of Company A is 3.1125. The grade is divided into 4 levels, which proves that there is still a certain gap between the asset management level of start-ups and mature companies. Finally, to find out the problems of the company's asset quality, the traditional financial analysis method is used to carry out a specific microanalysis of the evaluation indicators of its asset quality. In view of the existing problems, the following 5 rationalization suggestions are put forward: (1) invest cautiously and pay attention to the provision for asset impairment; (2) improve the efficiency of inventory operation and improve the use efficiency of idle funds; (3) keep up with the market demand to launch new products; (4) improve the quantity and quality of offline outlets and regularly check the sales situation; and (5) increase the proportion of intangible assets of companies, increase investment in R&D, and appropriately adjust the proportion of fixed assets. Due to the limited ability, the selection of evaluation indicators is not comprehensive enough, However, any financial data in the process of production and operation of an enterprise will have a certain impact on the asset quality, so the selection of indicators should be considered more comprehensively in the future research. By evaluating the asset quality of start-ups based on BPNN, it can help start-ups discover the gaps between them and mature companies to improve their asset management and enhance their asset management capabilities. This research has a certain reference for the application of AI technology in the asset management of start-ups.

The article "The Application of Artificial Intelligence Technology in the Asset Management of Start-Ups in the Context of Deep Learning" was published in 2022. Journal: Comput Intell Neurosci.

## Figures and Tables

**Figure 1:** The structure of BPNN.

**Figure 2:** The calculation process of BPNN.

**Figure 3:** The evaluation indicators system of asset quality.

**Figure 4:** The properties of evaluation indicator of asset quality.

**Figure 5:** Weights of evaluation indicators for mature companies in the same industry in 2019–2021.

**Figure 6:** The comprehensive score of asset quality of the five mature companies in the same industry in 2019–2021.

**Figure 7:** The standard of grading classification of the comprehensive score of asset quality.

**Figure 8:** Training results and training times of BPNN.

**Figure 9:** The original input data of the evaluation model of asset quality of Company A.

**Figure 10:** Comparison of asset existence.

**Figure 11:** Comparison of asset turnover.

**Figure 12:** The comparison of asset liquidity.

**Figure 13:** The comparison of asset profitability.

**Figure 14:** The comparison of asset structure.

## Data Availability

The data used to support the findings of this study are included within the article.

## References

[1] Lin J. Y., Cui W. H., Han B., Wang H., Liu X. H (2020). Research on additive manufacturing technology in the field of mold repair. *Materials Science Forum*.

[2] Peraka N. S. P., Biligiri K. P. (2020). Pavement asset management systems and technologies: a review. *Automation in Construction*.

[3] Ali M. R., Ratul M. R., Tisha R. T., Islam M. A (2021). A comparative performance evaluation of banking industry in Bangladesh: CAMEL rating approach. *International Journal of Financial Engineering*.

[4] Zheng Z. (2021). Energy efficiency evaluation model based on DEA-SBM-Malmquist index. *Energy Reports*.

[5] Cai X., Qian Y., Bai Q., Liu W (2020). Exploration on the financing risks of enterprise supply chain using Back Propagation neural network. *Journal of Computational and Applied Mathematics*.

The article "The Application of Artificial Intelligence Technology in the Asset Management of Start-Ups in the Context of Deep Learning" was published in 2022. Journal: Comput Intell Neurosci.

[6] Li Z., Ge Y., Su Z. (2020). Audience Leisure Involvement, Satisfaction and Behavior Intention at the Macau Science Center. *The Electronic Library*.

[7] Bukhsh Z. A., Stipanovic I., Saeed A. (2020). Maintenance intervention predictions using entity-embedding neural networks. *Automation in Construction*.

[8] Rezaei H., Faaljou H., Mansourfar G. (2021). Intelligent asset allocation using predictions of deep frequency decomposition. *Expert Systems with Applications*.

[9] Li Z., Li X., Tang R., Zhang L (2021). Apriori algorithm for the data mining of global cyberspace security issues for human participatory based on association rules. *Frontiers in Psychology*.

[10] Ioannou A., Angus A., Brennan F. (2020). Stochastic financial appraisal of offshore wind farms. *Renewable Energy*.

[11] Ma X., Guan Y., Mao R., Zheng S., Wei Q (2021). Modeling of lead removal by living Scenedesmus obliquus using backpropagation (BP) neural network algorithm. *Environmental Technology & Innovation*.

[12] Liu H., Liu J., Wang Y., Xia Y., Guo Z. (2021). Identification of grouting compactness in bridge bellows based on the BP neural network. *Structures*.

[13] Foscarin F., Rigaux P., Thion V. (2021). Data quality assessment in digital score libraries. *International Journal on Digital Libraries*.

[14] Sanchez-Segura M. I., Ruiz-Robles A., Medina-Dominguez F., Dugarte-Pena G. L (2017). Strategic characterization of process assets based on asset quality and business impact. *Industrial Management & Data Systems*.

[15] Alégroth E., Gorschek T., Petersen K., Mattsson M. (2020). Characteristics that affect preference of decision models for asset selection: an industrial questionnaire survey. *Software Quality Journal*.

[16] Franciosa I., Ferrocino I., Giordano M., Mounier J., Rantsiou K., Cocolin L (2021). Specific metagenomic asset drives the spontaneous fermentation of Italian sausages. *Food Research International*.

[17] Makropoulos A., Weir C., Zhang X. (2020). An analysis of the determinants of failure processes in UK SMEs. *Journal of Small Business and Enterprise Development*.

[18] Liu Z. (2019). Management of commercial assets in universities in the information age[J]. *International Core Journal of Engineering*.

[19] Villanti A. C., Vallencourt C. P., West J. C. (2020). Recruiting and retaining youth and young adults in the policy and communication evaluation (PACE) Vermont study: randomized controlled trial of participant compensation. *Journal of Medical Internet Research*.

[20] Piaskowska D., Tippmann E., Monaghan S. (2021). Scale-up modes: profiling activity configurations in scaling strategies. *Long Range Planning*.

The article "The Application of Artificial Intelligence Technology in the Asset Management of Start-Ups in the Context of Deep Learning" was published in 2022. Journal: Comput Intell Neurosci.

[21] Rastrollo-Horrillo M. A. (2021). Dismantling the myths about managerial (in)capabilities in micro-firms. SEAM intervention-research to develop management practices. *Scandinavian Journal of Management*.

[22] Shen T., Chang J., Xie J., Huang L (2020). Analysis of microchannel resistance factor based on automated simulation framework and BP neural network. *Soft Computing*.

[23] Yu Z., Qin L., Chen Y., Parmar M. D (2020). Stock price forecasting based on LLE-BP neural network model. *Physica A: Statistical Mechanics and Its Applications*.

[24] Yan Q. Y., Wang X. Y., He S. Q. (2012). Using transfer-entropy TOPSIS and BP neural networks model to early warning of external environments of life cycle asset management. *Advanced Materials Research*.

[25] Palau A. S., Dhada M. H., Bakliwal K. (2019). An Industrial Multi Agent System for real-time distributed collaborative prognostics. *Engineering Applications of Artificial Intelligence*.

[26] Meijer D., Scholten L., Clemens F., Knobbe A (2019). A defect classification methodology for sewer image sets with convolutional neural networks. *Automation in Construction*.

[27] Bangalore P., Patriksson M. (2018). Analysis of SCADA data for early fault detection, with application to the maintenance management of wind turbines. *Renewable Energy*.

[28] Ogunjo S. T., Adediji A. T., Dada J. B. (2017). Investigating chaotic features in solar radiation over a tropical station using recurrence quantification analysis. *Theoretical and Applied Climatology*.

